The article "Meta-Analysis and Data Mining-Based Study on the Expression Characteristics of Inflammatory Factors and Causes of Recurrence in Spinal Tuberculosis" was published in 2022. Journal: Comput Math Methods Med.

# Meta-Analysis and Data Mining-Based Study on the Expression Characteristics of Inflammatory Factors and Causes of Recurrence in Spinal Tuberculosis

**DOI:** 10.1155/2022/8246510

**Published:** 2022-09-22

**Authors:** Jun Wang, Shaoning Jiang

**Affiliations:** Orthopedics, Shanghai Public Health Clinical Center, Shanghai 250001, China

## Abstract

With the rapid development of modern medical information technology, hospitals are accumulating huge amounts of clinical data while providing medical services to patients, and in the era of big data, how to mine valuable information from the huge amount of clinical data so as to make new contributions to future disease diagnosis and medical research. In order to solve this problem, more and more scholars have introduced data mining techniques into the medical field in recent years, and mining and analysing medical data is a hot topic at present. If spinal TB is detected and treated early, not only can spinal deformities be prevented and treated but also the course of treatment can be shortened, the financial burden on the patient can be reduced, spinal function can be maintained, and eradication can be achieved without the need for surgical intervention. Early detection of spinal tuberculosis is the key to preventing and treating it. Therefore, in this paper, we use meta-analysis and data mining techniques to process and analyse the medical data of spinal tuberculosis disease, its main inflammatory factors expression characteristics, and the causes of patient recurrence.

## 1. Introduction

Tuberculosis of the spine is an infectious disease caused by Mycobacterium tuberculosis. Of these tuberculosis diseases, spinal tuberculosis is the most prevalent. According to the World Health Organization [1, 2], there are now approximately 9 million new cases of spinal tuberculosis worldwide each year, and approximately 1.5 million deaths from spinal tuberculosis each year [3]. In China, TB of the spine is the second most prevalent infection in the world, with the highest incidence in the country. Bone and joint tuberculosis is the most common form of spinal tuberculosis secondary to spinal tuberculosis, accounting for about 5-10% of cases, with spinal tuberculosis being the most common at about 50%. Spinal TB is most common in young people and occurs mainly in the lumbar spine, thoracic, cervical, and sacral spine. TB of the spine is a bony injury to the vertebrae that can easily lead to lesions that, if not treated promptly, can easily lead to spinal deformities and, in severe cases, affects the spine and compress the spinal cord [4]. Spinal nerve damage or paralysis occurs in 10% to 61% of patients with spinal TB.

There are four diagnostic bases for infectious spinal disease: symptoms, signs, specialist investigations, laboratory tests, imaging tests, and pathology [5]. The positive rate of blood cultures for brucella ranges from 10% to 74% (9), and the detection rate of Mycobacterium tuberculosis (TB) is 44.5% (10). Before the use of antimicrobial therapy, the positive rate of blood cultures is about 70%, and the positive rate of blood cultures is as high as 70%. The long cycle of blood cultures for brucella adds to the difficulty of early diagnosis [6–9]. The final diagnosis of spinal infection is established by puncture biopsy and surgical pathology, but surgical treatment is usually required. MRI is useful for the early diagnosis of infectious spinal lesions, assessing the extent of the lesion and the presence or absence of invasive intradural lesions, and visualising lesions in the spinal cord and nerve roots. It is currently the examination of choice for infected spinal lesions due to its better soft tissue resolution, multidirectional [10], multiparametric imaging, noninvasiveness, and clear visualisation of structures within the spinal canal. Therefore, exploring the expression characteristics and etiology of inflammatory factors in spinal tuberculosis is a useful reference for diagnosis, treatment, and prognosis.

## 2. Introduction to Relevant Theories

### 2.1. Medical Data Mining

Data mining is an interdisciplinary discipline that encompasses database technology, pattern recognition, machine learning, artificial intelligence, parallel computing, statistics, and data visualisation [11]. In short, data mining is the extraction of potentially valuable information and knowledge from large, incomplete, noisy, fuzzy, and random data of practical application. Data mining is an important part of knowledge discovery, which is based on a full and deep understanding of data, a high degree of abstraction and summary of the intrinsic and essential nature of data, and the sublimation of data from perceptual to rational cognition. Since it was introduced in the late 20th century, it has been valued by many experts and scholars [12].

The development of medicine has evolved from empirical medicine and experimental medicine to the current evidence-based medicine, which has a huge amount of medical data with characteristics such as objectivity and experimentation.

The process of medical data mining includes: problem definition, data preparation, data mining, result analysis, and knowledge application [13].

1. *Defining the problem*. First, a thorough communication with medical professionals is necessary to analyse their needs, define their requirements, determine their purpose, and measure their success
2. *Data integration*. Data integration (integrating different types of data from multiple archives or multiple repository operating environments), data purging (removing noisy and irrelevant data from the original data set, missing data, and removing dirt), data transformation (basically finding the characteristic representation of data, using transformation methods to reduce the number of valid variables or discovering data invariants)
3. *Data mining*. The main components are: selection of data models, determination of training and experimental processes, model building, model evaluation, etc. In order to verify the validity of the data mining and the correctness of the data, it is also necessary to verify the validity of the data in conjunction with clinical practice
4. *Research results*. The knowledge and rules found in data mining need to be judged as correct and easy to understand from the user's perspective. It is also important to evaluate whether the knowledge mined is medically meaningful, medically relevant, medically meaningful, and consistent with the original intent of data mining
5. *Use of theory*. The execution and control of the conclusions should be planned in detail, and a detailed summary of the whole project should be made and used in future medical practice

### 2.2. Introduction to Association Rules

The application of association rules in data mining is one of the most current concerns in data mining. Association rules are used to describe possible relationships between items of information in a database. The object of association rule mining is usually a transaction database, which was originally used in the retail industry, for example in supermarket sales management. The development of barcode technology has made it easier and better to collect data, so that huge amounts of transaction information can be stored, and association rules are used to identify customers based on their purchase behaviour. The information obtained through association rules can be used for catalogue design, merchandise layout, target marketing, etc.

The problem of association of item sets in customer transaction databases was first introduced by Agrawal et al. in 1993, and a typical Apriori mining method was introduced in 1994. Based on this, many scholars have explored association rules in depth. Their work is to optimise the existing Aprior algorithm, such as introducing random sampling, the idea of parallelism, and using hashing, in order to improve the mining efficiency of the algorithm; some have proposed a new method of association rule mining that is not related to Apriori, such as Jianwei et al.'s FP-Growth method and association rule mining based on association graph mining [14–17].

### 2.3. Meta-Analysis Theory

Meta-analysis is a statistical method for comparing and synthesising the same scientific questions. Combining all relevant studies allows for a more accurate assessment of the effectiveness of health care services compared to a single study and also helps to explore the consistency and differences between the results of different studies. And where different studies have different findings, meta-analysis can be used to produce a statistical analysis that is similar to the actual situation [18].

Meta-analysis mainly includes: (i) analysis of heterogeneity and statistical consistency tests on data from multiple independent experiments and (ii) evaluation of combined effects.

In meta-analysis, the test of heterogeneity is a very critical process, and the *Q*-test is mostly used to determine whether there is a significant difference in the heterogeneity of multiple independent studies, and it is usually considered that the results of each independent study are consistent at *P* > 0.1.

Effect values are generally selected based on the nature of the clinical study and the type of data. In meta-analysis [19], fixed-effects and random-effects models are usually used, with fixed-effects models being used where there is consistency across multiple studies, and random-effects models may be used to calculate different effect factors where different studies exist, for example, where different subgroup analyses are conducted and satisfactory results are still not obtained after heterogeneous analysis and processing.

Meta-analysis, especially based on high quality randomised controlled trials (RCTs), is considered to be a high level of evidence-based evidence which serves: (i) to achieve quantification; (ii) to address the same issues in a systematic and reproducible manner; (iii) to synthesise the same topics from multiple small samples to improve the statistical efficiency of the original results; (iv) to resolve inconsistencies in study findings and improve assessment of effects; (v) provide answers to questions not asked in the original study; (vi) explore the extent of publication bias in the existing literature; (vii) provide new topics for future research.

### 2.4. Theory of Spinal Tuberculosis

Spinal tuberculosis is a chronic disease with systemic pathology. Nationally, spinal tuberculosis is the most common, with spinal tuberculosis predominating and adnexal tuberculosis being very rare. In terms of location, the lumbar spine is the largest, followed by the thoracic spine. As for tuberculosis of the sacral and caudal spine, it is even rarer.

Classification of spinal tuberculosis:

Depending on the location of the lesion, it can be divided into two categories: the central type and the marginal type.

1. The central type of spinal tuberculosis occurs mostly within 10 years of age, mainly in the thoracic spine. Due to the rapid development of the tumour, the entire vertebral body is wedge-shaped and usually invades only one vertebra
2. Marginal spinal tuberculosis is predominant in adults, with the lumbar spine predominating. The intervertebral discs are damaged and the vertebral space is reduced. Cold abscesses develop first and then compression leads to spinal cord injury

Clinical features of spinal tuberculosis:

1. Systemic clinical manifestations include fatigue and weakness, loss of appetite, physical wasting, low fever in the afternoon, and vegetative dysfunction. Fever is common in children, and they do not like to play and cry at night
2. The early manifestation of pain is usually a dull ache. It is aggravated by walking and exertion and relieved by rest; the pain is aggravated by sneezing and coughing. The pain is mainly localized and radiating. Localised pain usually occurs on both sides of the spine or between the spinous processes and the spines. Following an injury, radiating pain can develop in the corresponding segmental innervation areas [20]. Patients with lesions in the thoracolumbar segment often present with pain in the lumbosacral region. If the lesion compresses the spinal cord and nerve roots, it can produce very intense pain that radiates outwards along the nerve roots. The pain is not very pronounced because of the distance between the spinal column and the spinous process: percussion is localised to the spinous process and there is pain
3. Disorders of posture. Due to differences in the location of the lesion, patients with cervical tuberculosis often hold their heads in their hands; patients with lumbar tuberculosis have back pain and are afraid to stoop when picking up objects
4. Spinal abnormalities, the most common being backward curvature of the spine. Posterior convexity is the most common type, with the spine bulging backwards at an angle. Children with thoracic spinal tuberculosis are prone to kyphosis because of the number of sites of their lesions
5. Myospasm, which is initially a reflex spasm of the muscles on the side of the spine due to pain, followed by spastic dystonia, leads to abnormalities in certain positions. Examples include cervical spondylosis in patients with tuberculosis of the spine and a self-expanding gait in patients with tuberculosis of the thoracolumbar segment. In children, the relaxation of the muscles after sleeping causes pain when turning over or changing position, resulting in “nocturnal crying in children”.

## 3. Application Method Design

### 3.1. Data Mining Model Construction

In the process of data mining, the expression characteristics of spinal tuberculosis inflammatory factor, the basic principles of relevance, feasibility, validity, and safety should be followed, and on the premise of satisfying the basic principles, the traditional method of generating the expression characteristics of spinal tuberculosis inflammatory factor is based on a simple inference system, while for multimorbidity users, this paper proposes that it is based on the original spinal tuberculosis inflammatory factor expression characteristics data. Based on the original spinal tuberculosis inflammatory factor expression characteristics data, this paper proposes to generate the final spinal tuberculosis inflammatory factor expression characteristics by data mining through association models to constitute an inference system for spinal tuberculosis inflammatory factors [21]. The model can also be used to mine the medical data of relapsed patients and to generate features on the causes of relapse. The model structure is illustrated in Figure 1.

One of the data mining processes is as follows:

1. *Stating the problem and clarifying the hypothesis*. In practical data mining, each project has its own area of expertise and application context, so it requires some understanding of the relevant expertise, business processes, etc. Thus, the analyst can understand the need and importance of the project. This process tests not only the analyst's technical skills but also the level of cooperation between the analyst and specific industry players [22]
2. *Data collection*. This step considers the generation and collection of data, and depending on the purpose of the data collection and the technical guidelines required, the extraction of data from the database is done to generate the data to be analysed. Usually, comprehensive, high quality, and accurate information is an important guarantee for data mining efforts. Mixed data and too much data will have a negative impact on the effectiveness and validity of data mining
3. *Data preprocessing*. After the appropriate information has been collected, it cannot be analysed directly. It must go through multiple stages of data preprocessing such as data cleaning, fusion, selection, and conversion. Since some problems are bound to arise during data collection, data cleaning is mainly to remove noise and inconsistency. Data integration is the process of bringing together various data resources, while data selection is the process of extracting relevant information from the data. Data conversion, on the other hand, is the process of merging and consolidating, making it possible to undergo conversion and uniform processing in order to form a format suitable for subsequent operations
4. *Data mining*. In practical engineering problems, methods more appropriate to the engineering context are used to solve them. This shows the role that appropriate algorithms play in the mining process. Firstly, the model is tested by selecting an appropriate data set to ensure its correctness and quality. And the appropriate modifications are made according to the actual situation.
5. *Data analysis*. The process of data interpretation is important. One is the impact of the knowledge models found in the data mining process on the value of the business; another issue is how to visualise the results of data mining. In addition, depending on the needs of the industry, there is a need to compare and analyse the results and conclusions obtained with the relevant industry knowledge, a field of knowledge that covers a wide range of topics, from the experience of experts to industry regulations. The performance of the finalised or general indicators assesses their effectiveness prospects.

### 3.2. Meta-Analysis Design

Data analysis was performed using the ReviewManager 5.3 software package. In the statistical data, the two categories of effective and ineffective and cured and uncured were expressed in terms of dominance ratio, relative risk, risk difference, risk ratio and HR, and in terms of weighted mean difference (WMD).

1. *Mapping the forest*. Meta-analysis focuses on the mapping and analysis of the forest map
2. *Testing for heterogeneity*. The primary means of testing is for tests where an *I*-value of more than 50% and a *P* value of less than 0.1 indicate heterogeneity and a random-effects model should be used. In contrast, for studies with good homogeneity, a fixed-effect model is usually used
3. *Tests of bias*. The “inverted funnel plot” is the current main mode of presentation. When there is bias, the point-shaped data on the curve is uneven
4. *Sensitivity analysis*. According to the JADAD scale, low quality and bias-causing literature was excluded, the remaining high quality literature was statistically analysed, and the two were compared to determine their stability

## 4. Application of Experimental Analysis

### 4.1. Introduction to the Data Set

The data were obtained from a medical case database developed by Cerner in the USA [23], and included hospital admissions of spinal TB patients from 130 hospitals across the country (2010-2020) over a 10-year period, including 18 in the Midwest, 58 in the Northeast, 28 in the South, and 16 in the West. This database contains 41 tables with 117 attributes. This database contains 740,366,643 medical records corresponding to 17,880,231 patients and 2,889,571 data provision sources.

The dataset includes more than 50 attributes, including the following characteristics:

1. This information is for inpatient cases
2. All are cases of spinal tuberculosis, which includes all types of spinal tuberculosis
3. The duration of hospitalisation ranged from 1 to 14 days
4. All tests performed in a laboratory setting
5. Details of all hospital medication administered were recorded
6. The dataset contains the following basic characteristics: patient number, race, sex, age, type of hospitalisation, length of stay, attending physician, number of clinical trials, glycated hemoglobin tests, diagnosis, number of drugs administered, number of treatments, number of hospitalisations, and number of emergency admissions in the year

### 4.2. Preprocessing of Spinal Nodule Data

ETL is a key part of the implementation of a data warehouse and undertakes the transformation from the data source to the destination data warehouse. The content of ETL focuses on the extraction, transformation, and loading of data to achieve structured data. The following are:

1. *Extraction*. The raw data is extracted from various commercial systems and used as a data source. Sixty-five tables with a total of over 800 fields were extracted from both clinical and research sources to construct a single disease-specific data marketplace for spinal tuberculosis.
2. *Transformation*. The extracted information was transformed according to preset rules, resulting in a consistent data format.
3. *Loading*. The transformed information is entered into the data warehouse as a source for later mining and analysis. In this paper, clinical information on spinal tuberculosis is processed based on the information process.

### 4.3. Inflammatory Factor Expression Characteristics Mining Analysis Results

The dataset includes medical records for each patient's length of stay in hospital, and changes in their attendance are important for the treatment of spinal tuberculosis. In this paper, we analyse the inflammatory response of patients in the context of hospital infection and look for the most common inflammatory expression factors in terms of inflammatory expression.

The following analysis of spinal TB coinfection will be completed using PAL, in the data preparation phase, as follows:

1. *Determine the storage procedure for the raw data to be analysed*. To temporarily store the results of all intermediate calculations, as opposed to the actual data tables that follow, create the table type storage procedure, see Figure 2.

(2) *Definition of metadata*. In the metadata table PAL_APRIORI_PAL_APRIORI_, the properties of each stored procedure using the association rule algorithm.

In PDATA_TBL, the inputs and outputs of the algorithm are identified in Table 1.

(3) *Definition of the results of the implementation*. The results of the implementation of the algorithm are placed in the output tables of the implementation results in Table 2 and the implementation results in Table 3.

The SQL statement is as follows: (a) drop table PAL_APRIORI_RESULT_TBL and (b) create column table PAL_APRIORI_RESULT_TBL (“PRERULE” VARCHAR(5000), “POSTRULE”VARCHAR(5000), “SUPPORT” Double, “CONFIDENCE” Double, and “LIFT” DOUBLE).

This resulted in four tables as shown in Figure 3.

#### 4.3.1. Implementing the Apriori Algorithm

Table 4 demonstrates the results of data mining for concurrent inflammation, which reveals a relationship between spinal TB and inflammation. The greatest proportion of granulomatous inflammatory factor expression features can be seen in the types of vertebral bone destruction and the greatest proportion of spreading granulomas in paravertebral lesions.

### 4.4. Analysis of Recurrence Cause Data Mining Results

Data mining of medical data revealed that 70.6% of patients had multiple spinal lesions which were extensive and jumpy and could not be completely removed. The patients were in poor physical condition with large spinal gaps, postoperative spinal instability, and poor circulation to the transplanted vertebrae, which can affect fusion and repair of the spine.

36.3% of relapsed patients relapse due to the unstable location of the spinal tuberculosis lesion. Postoperative fixation of the lesion is mainly internal and external to maintain the stability of the spine. The absence and destruction of the anterior midcolumn structures of the spinal cord during surgery for spinal TB lesion excision, bone graft fusion, and lesion removal results in poor spinal stability and severe retroconvex deformity, and spinal stability is a prerequisite for TB healing and bone graft fusion, and the final healing of spinal TB can only be achieved after the location of the spinal TB occurrence is stabilized.

In 40.7% of these relapses, irregular pre and postoperative chemotherapy caused the relapse, and irregular pre and postoperative chemotherapy is the main cause of spinal TB relapse. Therefore, appropriate chemotherapy before and after surgery is essential to prevent tumour recurrence and to ensure the success of surgery. Patients and families should therefore be informed of how to administer regular antituberculosis chemotherapy to prevent recurrence.

Conclusion: nutritional support, complete intraoperative excision of the lesion, close postoperative braking and pre and postoperative chemotherapy can effectively reduce and prevent postoperative recurrence.

### 4.5. Meta-Analysis Results

This meta-analysis was performed on 29 trials including 7,555 patients with a diagnostic threshold in the range of 7.0 to 14.2 Kpa. In data mining for inflammatory factors in spinal tuberculosis, a sensitivity of 0.84 (95% CI: 0.80 to 0.87), a combined specificity of 0.87 (95% CI: 0.84 to 0.89), a combined positive likelihood ratio of 6.3 (95% CI: 5.0 to 7.9), a combined negative likelihood ratio of 0.19 (95% CI: 0.15 to 0.23), SROC area under the curve was 34 (95% CI: 23 to 50), and SROC area under the curve was 0.92 (95% CI: 0.89 to 0.94). The statistical results of the spinal tuberculosis inflammatory factor data mining model are shown in Table 5.

1. The SROC curve is plotted as shown in Figure 4

(2) Forest mapping

As shown in Figure 5, there is a clear advantage in reducing spinal TB recurrence in cases where inflammation is well controlled.

(3) Sensitivity tests

Excluding one trial with a low Jadad score and reanalysing, the test of heterogeneity was *P* = 0.96 > 0.1, with good agreement, and using a fixed-effects model combined with effects analysis, 95% CI: 1.26 (1.12, 1.42), *P* = 0.0001, with no significant difference between the two, showing good stability. As shown in Figure 6.

## 5. Potential for Bias

An ‘inverted funnel plot' was drawn to see if there was any bias. The graph shows that the dotted distribution is not very symmetrical, representing a degree of bias as shown in Figure 7.

## 6. Conclusion

Data mining is an emerging discipline that has emerged in recent years. It makes comprehensive use of various learning methods and approaches such as statistics, rough sets, and fuzzy mathematics to extract abstract knowledge from massive amounts of data, thereby revealing the intrinsic relationships and essential laws of the objective world hidden in the data, thus enabling the automatic extraction of knowledge.

Spinal tuberculosis is one of the most common forms of osteoarticular tuberculosis, accounting for about 50% of all tuberculosis in the body, and is also a major cause of spinal deformity and paralysis. Due to its high rate of disability, it seriously affects the quality of survival of patients. Currently, surgery is the mainstay, but the recurrence rate of TB remains high in spinal TB surgery. Therefore, in this paper, data mining techniques were used to mine medical data in depth, and the data were screened and analysed. The most significant of these was found to be the expression characteristics of granulomatous inflammatory factors, and based on the information mined, the causes of recurrence were analysed and the incidence of multiple spinal lesions was found to be 70.6%. Meta-analysis of the various inflammatory profiles revealed a significant reduction in the recurrence rate of spinal tuberculosis with control of inflammation.

## Figures and Tables

**Figure 1:** Simple reasoning flow chart.

**Figure 2:** Stored procedure table.

**Figure 3:** Table of implementation results.

**Figure 4:** SROC Plot.

**Figure 5:** Forest map of recurrence.

**Figure 6:** Medium sensitivity test.

**Figure 7:** Inverted funnel diagram.

**Table 1:** Parameter settings for PAL_APRIORI_ PDATA_TBL.

ID	Typename	Direction
1	DISEASE.PLA_APRIORI_DATA_T	In
2	DISEASE.PLA_CONTROL_T	In
3	DISEASE.PLA_APRIORI_RESULT_T	Out
4	DISEASE.PLA_APRIORI_PMMLMODEL_T	Out

**Table 2:** Structure of the implementation results data sheet.

Serial number	Field	Data type	Description
1	PRERULE	VARCHAR(500)	Frequent items
2	POSTRULE	VARCHAR(500)	Item ID
3	SUPPORT	DOUBLE	Support
4	CONFIDENCE	DOUBLE	Confidence

**Table 3:** Structure of the data sheet for the implementation result parameters.

Serial number	Field	Data type	Description
1	ID	INT	Frequent items
2	PMMLMODEL	VARCHAR(5000)	Item ID

**Table 4:** Data mining results for the dataset.

Variables	BS(*n* = 40cases)	NPS(*n* = 1case)	TBS(*n* = 6cases)	*χ* ^2^	*P*
Epidural abscess-characteristic 1				2.790	0.248
Absent	39(36.11%)	16(14.81%)	53(49.07%)		
Yes	1(10.00%)	2(20.00%)	7(70.00%)		
Type of vertebral bone destruction-characteristic 2				38.856	0.001
Granuloma	28(63.64%)^a^	9(20.45%)^a^	7(15.91%)^b^		
Confined abscess	11(19.30%)^a^	8(14.04%)^a,b^	38(66.67%)^b^		
Lytic abscess	1(5.88%)^a^	1(5.88%)^a,b^	15(88.24%)^b^		
Paravertebral lesion-feature 3				45.630	0.001
Restricted granuloma	22(62.86%)^a^	7(20.00%)^a^	6(17.14%)^b^		
Spreading granuloma	2(66.67%)^a^	0(0.00%)^a^	1(33.33%)^a^		
Confined abscess	15(32.61%)^a^	10(21.74%)^a^	21(45.65%)^a^		
Spreading abscess	1(2.94%)^a^	1(2.94%)^a^	32(94.12%)^b^		

**Table 5:** The statistical results of the spinal tuberculosis inflammatory factor data mining model.

Main parameters	Slight inflammation		Significant inflammation	Severe inflammation	Early spinal tuberculosis			
	Point 95% CI estimate		Point estimate	95% CI	Point 95% CI estimate		Point estimate	95% CI
SEN	0.80	0.71-0.87	0.84	0.81-0.86	0.87	0.84-0.89	0.89	0.87-0.91
SPE	0.76	0.69-0.82	0.77	0.72-0.80	0.84	0.80-0.87	0.89	0.86-0.92
PLR	3.90	2.60-5.80	4.70	4.0-5.5	6.3	5.0-7.9	8.2	6.6-10.1
NLR	0.30	0.23-0.37	0.28	0.23-0.34	0.19	0.15-0.23	0.12	0.09-0.16
AUC	0.85	0.82-0.88	0.88	0.84-0.90	0.92	0.89-0.94	0.95	0.93-0.97
DOR	13.008.00-21.0017.00		12.00-23.0034.00		23.00-50.0067.00			44.00-101.00

## Data Availability

The dataset used in this paper are available from the corresponding author upon request.
